The article "Analysis of the Questioning and Dialectical Relationship between the Pursuit of Intensity in School Physical Health Education" was published in 2022. Journal: J Environ Public Health.

# Analysis of the Questioning and Dialectical Relationship between the Pursuit of Intensity in School Physical Health Education

**DOI:** 10.1155/2022/7433428

**Published:** 2022-10-06

**Authors:** Shuli Yuan

**Affiliations:** ZhengZhou University of Technology, Zhengzhou 450000, China

## Abstract

In the rapid development of the country and schools, physical education and health programs have gradually become an essential part of schools in order to improve students' core physical education skills and literacy, and have a very important role and impact on students' physical and mental health development. The school P&H program not only conveys to teachers and students the knowledge and training skills to improve school sports and enhance physical fitness but also fully develops the awareness and ability of teachers and students to work hard and collaborate with each other. This paper examines and analyzes the problems and dilemmas associated with the pursuit of health and sport-specific intensity in school sports and combines theories of health and exercise, physical education, training, and moral education through literature review, logical analysis, and value analysis. The purpose of this paper is to clarify the different logics and orientations of specific sport intensity regulations, school sport health pursuits, and school sport teaching and to clarify and correct related issues, so as to provide theoretical and practical support for school sport to better implement the concept of “health first” and further promote school sport reform and sound development. In this paper, we analyze the relationship between exercise and health in physical education programs of teachers and schools from the perspective of natural dialectics and find out some outstanding problems that may exist in them, so as to effectively promote the development of students' physical and mental health.

## 1. Introduction

### 1.1. Health Education

Health education, as we are promoting it, is an education that requires the transmission of health knowledge to students and the establishment of hygienic behaviors, while making environmental improvement a central part of the education [1]. The reason why we are promoting health education in schools is to enable people to have healthier lifestyles and behaviors, so that through each individual's improvement, the health of society as a whole can be improved. Health education, fundamentally, is an educational promotion and intervention activity that allows people to have a healthier philosophy through purposeful intervention in schools, so that they can have healthier behaviors and habits, which will enable them to prevent diseases, then, improve their physical and mental health and finally improve their quality of life as shown in Figure 1.

Currently, there is no clear definition of the concept of health education. In China, the concept of health education refers to the planned educational and social activities organized by health education-related departments to disseminate health-related knowledge, strengthen people's health awareness and concepts, and promote the conscious adoption of health-friendly lifestyles and behavioral habits.

Tomokawa et al. mentioned that the World Health Organization considers health education as a way to better guide people to adopt health-friendly behaviors [2]. Health education is a way to better guide people to adopt healthful lifestyles by inducing and encouraging them to do so. People can take the initiative to understand and value health, and then maintain their own health. People learn to use existing resources and facilities in a rational way to improve their health. Martinsen viewed health education as a science to help people change unhealthy behaviors and establish healthy behaviors to achieve the purpose of promoting people's health [3]. Its research includes health knowledge, technology, education, and intervention methods, involving various disciplines such as education, psychology, sociology, and behavioral science. According to Huang et al., health education is the dissemination of health care knowledge and skills to people and the influence on their cognitive attitudes and values. It cultivates people's health awareness, positive attitude towards society and the ability to maintain their own health, and motivates them to actively implement health-friendly lifestyles and behaviors to reduce the influence of risk factors.

### 1.2. Physical Education Instructional Design

Physical education is a complex collection of teaching phenomena, which is a purposeful and organized process of teaching by teachers and students according to certain plans and curriculum standards, called physical education. In view of the increasing trend of deepening the reform of school physical education curriculum in China, the process of scientific research and planning to optimize the work according to different teaching purposes and conditions is physical education teaching design. The complete physical education design involves such aspects as making a reasonable teaching plan, designing a teaching mode suitable for students' physical and mental characteristics, and using teaching equipment and devices as shown in Figure 2.

### 1.3. PRECEDE Model Theory

The core of the PRECEDE model is the educational organization diagnosis, which consists of three important influences: dispositional factors, contributing factors, and reinforcing factors [4]. The dispositional factors, which usually precede the occurrence of a behavior, are the motivation, desire, or factors that induce a behavior, such as knowledge, attitude, or beliefs. The health education knowledge rate is a survey of the existing health education knowledge of physical education teachers and students to detect the current level of knowledge of physical education teachers and students in Kaifeng urban high school health education module. In addition, students' knowledge and attitude toward health education determine the quality of health education they receive, and the importance of health education by school leaders is an important guarantee for health education implementation. In this study, the awareness rate of physical education teachers and students about health education and the knowledge of physical education teachers, students, and supervisors about health education were taken as the tendency factors for implementing health education modules as shown in Figure 3.

## 2. Description of the Probiem

### 2.1. Problems of Health Education in School Sports

#### 2.1.1. Formalization of Health Education Process

Health education is not only the education of basic health knowledge but also the combination of acquired education and nurturing education [5]. The nurturing nature of health education in school physical education means that students should gradually improve their health and develop regular health behaviors through physical education courses and in their daily lives; only when students have a correct understanding of health will they form an awareness of the importance of sports, and only when students have an understanding of the importance of health will they form a health consciousness or a sense of participation in sports and will actively participate in sports activities [6]. Therefore, the subjects of health education are not able to deeply understand the inner relationship between these three levels, which leads to the formalization of the process of health education for students in the practice of physical education. The acquired nature mainly refers to the teaching of basic health knowledge through physical education, and the latter is the object of focus in school physical education. The latter is the focus of physical education in schools. In reality, the main body of health education in school physical education understands health in the process of teaching practice as promoting students' health as long as they participate in sports, which is a superficial understanding, not that students can be formed by participating in sports, but involves students' understanding of health, students' health awareness, and students' health behavior.

#### 2.1.2. Lack of Clear Direction for Aid Health Education

School sports cannot take all the responsibility of health; physical education as the core part of school sports is the implementation of sports-related health education through the teaching of sports programs and some indoor health education classes [7]. So, what are the health education goals? However, the complexity of the content and the emergence of health knowledge not related to physical education make the health education in physical education generalized, such as understanding the danger of drugs to individuals, families, and society, and the health education in the general high school physical education and health curriculum standard proposes to understand the risks of Internet dating and to understand the risks of AIDS and other diseases. For example, in the health education in the general high school physical education and health curriculum, it is suggested that understanding the risks of online dating and understanding infectious diseases such as AIDS and tuberculosis could be more appropriately covered by nonphysical education courses in school [8]. The content of health education listed in the curriculum standards is undoubtedly correct, but some health knowledge that is not directly related to physical education can lead to a generalization of health education goals, resulting in a lack of clear goal guidelines for health education.

### 2.2. The Current Situation of Integration of Physical Education and Health Education

As shown in Figure 4, due to the specificity of the current educational background in China, there is no template for the integration of physical education and health education, and there is only a genuine physical education and health teaching model with Chinese characteristics that can be developed in conjunction with the current teaching level.

There is not enough time to teach the theory of the curriculum, and some schools do not even teach the basic theory of classroom teaching to students; most of the physical education equipment in schools are various kinds of physical education equipment needed to teach physical education skills, and the area of sports fields that can be used is small. These factors limit the development and teaching of physical education and health courses.

Education administration departments at all levels have yet to improve their knowledge of “physical education” in their teaching work, and health education accounts for a smaller proportion of the practical teaching activities in physical education [9]. Knowledge and skills to carry out health education, school physical education workers have not established a modern view of health integrated with social development, and many schools' training personnel specialties have not become a training base for training health education, and the integration of physical education and health education has not yet attracted the attention of the whole society.

### 2.3. Problems in the Integration of Physical Education and Health Education

#### 2.3.1. Insufficient Attention to Work

Teachers' knowledge of physical education and health education, parents' ideological perception of physical education and health education, and students' curricular understanding of physical education and health education all constrain the development of physical education and health education. At the same time, students do not pay attention to health education, their half knowledge of health education and weak health consciousness, which invariably affect the development of students' physical health [10]. We should strengthen the ideological awareness of students, carry out the popularization of health education knowledge, and also strengthen the relevance of the physical education curriculum to the standards, popularize students' health education, promote the importance of health education, improve students' awareness cognition of physical exercise, and improve students' physical fitness test scores. Physical education and health education are mutually collaborative and codeveloping, strengthening the integration and development between physical education and health education, forming a systematic and interpenetrating teaching arrangement, and promoting students' physical fitness and health development as shown in Table 1.

#### 2.3.2. Management Mechanism Is Not Perfect

The integration of physical education and health education in China needs a longer-term development to achieve a higher level of connection [11]. The government's education administration department has not formed a more systematic and standardized guidance system for the development of physical education and health education and lacks the knowledge of physical education and health education in theoretical integration. For this course is the lack of teaching, lack of assessment, lack of supervision phenomenon, the integration of physical education and health education should establish a sound management organization, improve management regulations and systems, and effective evaluation and supervision system. Integrate social resources, strengthen the links with social welfare organizations, and invite students' parents to participate, so as to create an evaluation and supervision system that combines school, society, and parents to better develop physical education and health education.

## 3. State of the Art

### 3.1. Low-Intensity Characteristics of Physical Education Process

From the definition and composition of teaching, it includes two parts: “teaching” and “learning” [12]. In addition to general teaching, physical education also highlights the teaching of skills (mainly techniques) in each sport, with the specific focus on “teaching” and “learning” of skills and “practice” and “competition” throughout. This is also the basic way of teaching physical education in primary and secondary schools, which is usually referred to as a “new lesson” (or new content) [13]. This is also an adaptation to the current requirements for teaching multiple sports in primary and secondary schools, the basic level of most students, and the fact that it is difficult for most students to learn and master many sports in a limited number of class periods (except for options and special improvement classes). In the teaching cycle, only some sports, such as basketball and soccer, students only learn single or partial techniques to compete and reach a high level of athletic intensity in chasing and grabbing (even then, such sports should not emphasize athletic intensity at the expense of learning and improving each technical aspect). For many sports, especially those that are technically difficult or require a high degree of technical articulation, the main task, content, and important feature of physical education is the gradual mastery and proficiency of skills through a relatively low-intensity teaching, learning, and practicing process. If students do not learn progressively, it will be difficult for them to complete the subsequent complete technique or have some negative consequences as shown in Figure 5.

In terms of the specific arrangements for technical learning, some individual sports are subject to constraints such as single exercise intensity, technical difficulty, safety, space, and teaching organization, so students need to rotate through the exercises in a sequence [14]. For reasons of necessary learning observation, attention maintenance, interval rest, safety, etc., it is not appropriate to arrange other or excessive physical activities during many rotations, which will also lead to a decrease in the intensity and density of exercise in a single period. First, during individual student practice, the teacher may provide individual instruction, protection, or assistance, while other students observe or learn. Second, because technology learning is different from physical practice, students' learning of a particular technology in a given unit of instruction should be integrated and continuous, and their attention should be focused on the specific learning task for a long period of time without frequent interruptions and distractions from other irrelevant stimuli and information. Again, breaks in practice are a necessary rest and recovery [15]. Therefore, even if there are sufficient venues and equipment, it is not advisable to increase the intensity and density of exercise through other physical exercises or excessive group exercises during the rotation of the technique learning and improvement phase, otherwise, the teaching process of specific techniques will be fragmented and fragmented, or not conducive to students' physical recovery, thus reducing the effectiveness of learning and practice. For example, the intensity of single exercises is high for events such as box jumps, vaulting, single and double bars, and throwing, etc. The process of waiting in line after the exercises is not only a time to rest and recover but also a process to observe and listen to the teacher's comments and experience other people's technical movements. In addition, for some events, it is not advisable to schedule other exercises during the rotation (to increase intensity) for safety reasons.

### 3.2. The Way to Develop Moral Education Based on Physical Education

The reason why “physical education” is different from “sports” and “physical activities” is largely due to the fact that moral education can be consciously infiltrated in physical education. Compared with other courses, physical education has a more prominent “literacy” moral education value. As an important part of school education, physical education should not be self-relegated to mere sports and fitness activities. However, in order to increase the intensity and density of sports, the “noneffective sports” time of physical education classes is being consciously compressed, and the moral education contents and elements in them are also unconsciously ignored and excluded.

As far as the development of moral education activities in physical education is concerned, it has little to do with intensity or is mainly characterized by low intensity [16]. First, in terms of the composition of moral education-related qualities (e.g., physical education moral character), it involves elements of knowledge, emotion, intention, and action, of which only “intention-will” is directly (and not necessarily) related to high-intensity sports. Second, in terms of the content of moral education, it includes political, ideological, moral, and psychological aspects, except for some psychological qualities that can be strengthened by some high-intensity sports, others such as rules, aggressiveness, and cooperative spirit are related to different programs and not necessarily related to intensity, while ideological and political aspects are not even related to sports. Moral education in physical education can be divided into sports-related character and general social character, the latter involving, for example, classroom routines, discipline education, and other nonsports, intensity elements in the teaching interaction. Thirdly, from the viewpoint of moral education methods, including encouragement, praise, criticism, guidance, persuasion, case education, and typical education, all of which are mainly related to the use of language and need to be carried out in conjunction with various times of physical education, such as before, during, between, and after sports. Some practical activities of moral education also need to be penetrated with the help of various kinds of colorful and diverse nonintense activities. Fourth, from the distribution of moral education value, many low-intensity projects and low-intensity projects in unit time, such as martial arts, extended sports, track and field, gymnastics, games, and other activities, have unique moral education value. Fifth, in terms of the transformation of sports moral character to social moral character, some of the moral values embedded in sports programs, if they are only spontaneously participated by students, are more reflected in the sports context, while to transform into social character beyond specific sports, teachers still need to consciously conduct nonsports educational guidance. These moral education activities are either not related to intensity or occur more often in low-intensity teaching (sports) scenarios or even in “noneffective sports” time, as shown in Figure 6.

### 3.3. Analysis of the Effect of Integrating Health Education into Secondary School Physical Education

According to the physical health status of the students in the two classes before the experiment (Table 2), we can conclude that the physical health score of the boys in the experimental class (70.45) before the experiment was better than that of the boys in the control class (67.43), and the *T* value was -1.476, and the *P* value was 0.143, indicating that there was no significant difference in the physical health scores of the boys in the two classes before the experiment at the 5% significance level. The mean physical fitness score of girls in the experimental class before the experiment was 76.43, while that of girls in the control class was 73.21, and there was no significant difference between them at the 5% level of significance (*T* = −1.646 and *P* = 0.104). This shows that there is no significant difference between the physical fitness scores of male and female students in the experimental and control classes before the experiment and the randomness of the experimental class sampling [17].

According to the table of physical health status of students in the two classes after the experiment (Table 3), we can conclude that the physical health score of male students in the experimental class after the experiment was 77.38 and that of male students in the control class was 70.07, and the *T* value was -3.476, and the *P* value was 0.000, indicating that there was a significant difference between the physical health scores of male students in the two classes after the experiment at the 5% significance level. The mean physical fitness score of the girls in the experimental class was 80.96 and that of the girls in the control class was 75.83, and the *P* value was much less than 0.05, indicating that there was a significant difference between them (*T* = −2.95 and *P* = 0.004). It can be seen that the physical fitness scores of both male and female students in the experimental and control classes improved after the experiment, but in terms of absolute values, the experimental class improved more than the male and female students, indicating that the implementation of the “Health + Physical Education” teaching mode probably had a positive effect on students' physical fitness.

### 3.4. Low-Intensity Programs Based on Physical Education Unit Periods

In contrast to the specific intensity requirements, the following types of sports (complete practice and even game sessions) exhibit relatively low average intensity characteristics during the instructional unit periods (within a given practice or game time) [18].

- Short duration and high intensity-long interval programs. In terms of each practice, this type of program is more intense but not longer in duration. Due to the higher intensity, longer intervals and recovery time are required between multiple practices or games. In between each practice or competition, it is advisable to arrange rest or low-intensity activities; if there is not enough interval time for such projects, students will not only fail to play at the proper level but also damage the technical form and may easily lead to injury. Related events mainly include athletics (such as high jump, long jump, sprint, middle run, etc.), swimming and other physical events as well as gymnastic events that favor physical fitness (such as vaulting, box jumping, goat jumping, etc. that require running assistance) [19]. This interval and rhythm are determined by the characteristics of these programs (it is not advisable to arrange other exercises or sports of higher intensity during the interval), and they may be at a lower average intensity and density level during the unit period
- Continuous low-intensity program. These programs are of lower intensity and longer duration and can be maintained at a lower intensity for a longer duration, such as yoga, archery, shooting, taijiquan (noncompetitive routines), curling, air bamboo, some unarmed (apparatus) gymnastics, and specialized jogging. For example, the more skilled the practitioner, the lower the average heart rate level during practice. The average heart rate during practice (including multiple practice sessions) was about 126 beats/min, 110 beats/min, and 95 beats/min for general college students, professional students, and skilled adults, respectively

These programs not only have unique sporting, humanistic, and educational values but also their health values, as different forms of sports should not be neglected, either in terms of promoting physical and physical health indicators or in terms of promoting psychological and social health. For example, short-time, high-intensity, and long-interval programs emphasize physical fitness, while low-intensity programs such as taijiquan and yoga have a wide popular base, and their health value has been confirmed by modern science. Although some of these programs have not yet been widely promoted and popularized in schools, the relevant systems, policies, and requirements should leave room for their expansion.

## 4. Results Analysis

### 4.1. Considerations for Exercise Intensity Requirements and Application

School physical education has multidimensional values, goals, and inherent regulations, and different content may have different intensity requirements, even independent of intensity, and it is not appropriate to uniformly implement solid physiological-exercise intensity requirements or indicators (e.g., it is not appropriate to use this as a uniform requirement for the entire class or each class). The intensity requirements should take into account the sport, physical education, and humanistic values to reflect different teaching goals, rhythms, and styles. Even for the pursuit of health, it should go beyond its association with a specific intensity and be related to the multidimensional composition of health and the type of exercise [20].

The following factors should be taken into account when determining the intensity of sports in physical education: first, the intensity of a particular sport is usually associated with a sport competition, and it is important to prevent the intensity of the competition from interfering with skill learning or destroying the rules of the sport and to prevent the selection of high-intensity competitions. It should not be generalized or overused to increase intensity and should be considered in the context of its application. Second, intensity requirements in specific exercise situations should not be based on “low and high” intensities and “all” averages, but should be “appropriate” and individually tailored. Third, in the sense of “healthy” pursuit and “appropriate” intensity, the requirement of specific average (medium-high) intensity is more applicable to physical education activities and physical education classes or parts of classes in which the intensity varies in a certain appropriate range, so it should be more. The requirements should be used as an optional model or in specific contexts. Accordingly, physical education should not be pursued as a “comprehensive class” associated with intensity, thus diluting the distinction between the different objectives, tasks, and content of the class, or even falling into a solid pattern.

### 4.2. Improving Physical Education Teachers' Health Education Competence in Multiple Ways

The realization of the weakened health education function of physical education requires physical education teachers to have health education ability, which requires attention to three kinds of ability: first, the ability to design and teach health knowledge, which is the ability of physical education teachers to design basic knowledge such as infectious diseases, reasonable diet, and safety and risk avoidance based on the content of health education, and to design and organize it using network and multimedia means to teach students; second, the ability to generate health education content during the teaching of motor skills, which is part of the implicit psychological and social adaptation ability of health education [21]. The second is the ability to generate health education content in the process of teaching motor skills. Part of health education is the implicit content of psychological and social adaptability, which is formed through students' participation in sports learning, student cooperation, and team dialogue. The teacher should encourage the students if they can actively complete the exercise, and if they have to give up, the teacher should actively intervene with the students to regulate their psychological state, as in Figure 7. Third, the ability to integrate health content across disciplines, health education has content beyond physical education itself; physical education teachers need to selectively integrate the content of other disciplines related to it to enrich the teaching content, such as the integration of physical education and physiological health class related knowledge, through the form of indoor physical education theory class to explain to students the impact of physical education on physiological health.

### 4.3. Implementing Health Education Teaching Using Different Teaching Methods

Different health education teaching methods are used for different types. One is indoor health education class; the content of the explanation is based on the health knowledge that students better grasp and understand, such as the haze weather awareness of sports protection measures, the impact of the environment on students' sports, the harm of bad emotions on the human body, how to carry out a reasonable nutritional diet, etc., the teaching of health knowledge that is based on students' understanding and awareness. The second type is the health education teaching in skills teaching, focusing on students' physical health, mental health, and the cultivation of physical exercise awareness and habits, focusing on creating a variety of physical education learning situations to shape students' physical and mental experiences, simulating scenarios of students' sports injuries for physical education teachers to demonstrate scientific methods of dealing with injuries, so that students have a more intuitive understanding of the handling of that sports injury; the third category is the cooperation with school medical and nursing forces, or the establishment of cooperative relationships with professional medical and nursing forces outside the school. The third type is to cooperate with the school's medical forces or establish a partnership with professional medical forces outside the school, so that professional medical forces can be incorporated into the health education for students. For those operational and professional health knowledge such as artificial respiration and cardiopulmonary resuscitation, the teaching of professionals is more convincing and intuitive, and will deepen students' understanding and application of health knowledge.

## 5. Conclusions

The dialectical relationship between sports and health and the practice of dialectics tell us that everything should have certain two sides, to use the dialectical scientific eye to correctly view the problems that exist and to correctly understand and view the health of school sports, which bring teachers and students a variety of benefits and its drawbacks. The same is true for school sports. Properly conducted sports greatly promote the development of students' physical and mental health, but in any case, without a rational use of scientific methods to conduct sports, there is a risk of unnecessary psychological damage to students. Using the scientific dialectic of nature accurately analyzes all the relationships between sports and health, proving that the relationships between all things are interconnected, constantly changing, and developing, and that correct scientific judgments can be made in practice, so that new scientific methods or new means can be adopted to guide students in various sports, improving the psychological and physical qualities of students, and achieving the physical and psychological well-being of teachers and students' overall healthy development. In the future, the integration of health education into secondary school physical education will be beneficial in promoting students' health knowledge and helping them to develop healthy behaviors, with a more significant impact on students' eating habits in the short term, while the impact on their lifestyle habits may require more sustained intervention.

## Figures and Tables

**Figure 1:** No disease and health.

**Figure 2:** Flow chart of instructional design.

**Figure 3:** PRECEDE model theoretical architecture.

**Figure 4:** Curriculum model development research hotspots.

**Figure 5:** Dimensional relationship of school physical health education scale.

**Figure 6:** Physical education curriculum model development pathway map.

**Figure 7:** Ways to integrate health education in campus physical culture.

**Table 1:** Classroom teaching model concept of physical education combined with health education.

Lesson module	Design content	Design ideas
Preparation activities	Explain the significance of doing warm-up activities before exercise	Health education is included in the preparation activities section, the basic section, and the ending section.
Basic section	Basic theoretical knowledge such as rules and developmental functions is taught according to sports	
Closing section	Explaining the role of postexercise relaxation activities	

**Table 2:** Comparison of students' physical fitness scores in the two classes before the experiment.

	Experimental classes	Control class	*T* value	*P* value
Male	70.45 ± 8.747	67.43 ± 11.782	-1.476	0.143
Female	76.43 ± 8.785	73.21 ± 11.141	-1.646	0.104

**Table 3:** Comparison of students' physical health scores in the two classes after the experiment.

	Experimental classes	Control class	*T* value	*P* value
Male	77.38 ± 8.896	70.07 ± 11.055	-3.647	0.001
Female	80.96 ± 7.435	75.83 ± 9.581	-2.95	0.004

## Data Availability

The labeled data set used to support the findings of this study is available from the corresponding author upon request.
